RETRACTED

# Mechanism of Pilose Antler in Treatment of Osteoporosis Based on Network Pharmacology

**DOI:** 10.1155/2022/5298892

**Published:** 2022-03-30

**Authors:** Baoshan Liu, Aifei Wang, Zihou Cao, Junjie Li, Miao Zheng, Youjia Xu

**Affiliations:** ^1^Department of Orthopaedics, The Second Affiliated Hospital of Soochow University, Suzhou 215004, China; ^2^Institute of Osteoporosis Diagnosis and Treatments of Soochow University, Suzhou 215004, China; ^3^Osteoporosis Clinical Center, The Second Affiliated Hospital of Soochow University, Suzhou 215004, China

## Abstract

**Background:**

The purpose of this study was to demonstrate the pharmacodynamic material basis and molecular mechanism of pilose antler (PA) in the prevention and treatment of osteoporosis (OP) by the method of network pharmacology.

**Methods:**

First, the active components of PA were screened by BATMAN-TCM database, and the component targets were obtained from the SwissTargetPrediction online tool. Moreover, the relevant target genes of OP were obtained by searching the DisGeNET database. Second, the Venn diagram was drawn to obtain the PA-OP common targets, and the protein-protein interaction (PPI) network and drug-component-target (D-C-T) network were constructed by Cytoscape software. Finally, the GO functional annotation and KEGG pathway enrichment analysis of common targets were performed using the Metascape online tool.

**Results:**

82 common targets were identified by generating a Venn diagram. The PPI network of 82 common targets indicated that the top 5 nodal targets, including PIK3CA, MAPK1, ESR1, AKT1, and SRC, were strongly associated with other proteins. The D-C-T network suggested that the active components with high degree of connectivity include Prostaglandin E1, 17-Beta-Estradiol, Alpha-Estradiol, and Estrone. Furthermore, the GO enrichment analysis revealed that the biological process categories were dominated by response to peptide, cellular response to lipid, regulation of MAPK cascade, and so on. Additionally, the KEGG pathway analysis indicated the estrogen signaling pathway, osteoclast differentiation, and HIF-1 signaling pathway might have critical effects on the development of OP.

**Conclusion:**

The study shows that PA has the characteristics of multi-component, multi-target, and multi-pathway in treating osteoporosis.

## 1. Introduction

Osteoporosis (OP) is a highly prevalent disorder characterized by low bone mineral density and an increased risk of fracture [1, 2]. Osteoporotic fracture becomes increasingly common in women after 55 years of age and men after 65 years of age, resulting in substantial bone-associated morbidities and increased mortality and healthcare costs [1]. Therefore, effective treatment of OP is necessary. Recently, there are substantial advances in the availability of a range of drug treatment for OP, such as bisphosphonate, RANK ligand inhibitor, estrogen, selective estrogen receptor modulators, and parathyroid hormone receptor agonist [1]. However, when used in high doses or for long periods of time, these drugs may lead to side effects such as gastrointestinal reactions and acute renal failure. Therefore, it is necessary to find potential drugs with significant efficacy and high safety for the treatment of OP [3].

RETRACTED

Chinese traditional medicine has a good effect in treating OP, and it has few side effects. Pilose antler (PA) is the only completely regenerable tissue found in mammals and has extremely rapid growth rates (∼1.7 cm/day in red deer) [4, 5]. PA is commonly used in clinical Chinese medicine because of its beneficial effects on chronic inflammation and oxidative injuries, which can protect human organs, including the brain, lungs, and liver [6, 7]. Some studies have indicated that PA has a protective effect against OP due to kidney deficiency, which is a traditional Chinese medical term, mainly referring to the insufficient essence and poor qi of kidney [8]. Moreover, it plays a significant role in bone and tissue repair and health improvement; both deer antlers and human bone develop via intramembranous and endochondral modes of ossification [9]. Chunhui et al. reported that PA protects osteoblasts from oxidative injury through EGF/EGFR signaling [6]. Liu et al. demonstrated that PA can promote osteoblast differentiation and block TNF-*α*-mediated suppression of osteoblastogenesis in vitro via the NF-kB/p65 pathway as well as inhibit osteoclastogenesis in vitro [10]. However, due to the multi-component nature of Chinese medicine, its mechanism of action is still unclear.

In 2007, the concept of “network pharmacology” was systematically expounded by pharmacologist Hopkins in Nature Biotechnology for the first time, which integrates many new cross-disciplines such as systems biology and bioinformatics [11]. Network pharmacology was mainly used to discover all candidate targets, functions, and mechanisms of bioactive compounds for the treatment of disease [12]. In this study, we use the method of network pharmacology and construct a drug-component-target (D-C-T) network to explore the possible molecular mechanism of PA in the treatment of OP.

## 2. Materials and Methods

### 2.1. Screening of Active Components of PA

The active components of PA were acquired from BATMAN-TCM (https://bionet.ncpsb.org/batman-tcm/index.php) [13] by inputting “pilose antler” into the search box, and oral bioavailability (OB > 30%) and drug similarity (DL > 0.18) were set as the two key ADME indexes. Afterwards, the components were input into PubChem (https://pubchem.ncbi.nlm.nih.gov/) [14] to collect the chemical structures, SMILES, and the required parameters for target prediction.

RETRACTED

### 2.2. Target Identification of PA

In the present study, the component targets were obtained from SwissTargetPrediction (https://www.swisstargetprediction.ch) [15], which is an online tool that allows you to estimate the most probable macromolecular targets of a small molecule, assumed as bioactive. In brief, the potential target prediction was performed by inputting active components into SMILES with the organism limited to “*Homo sapiens*” and high probability targets (probability > 0).

### 2.3. Search of OP-Related Targets

OP-related targets were obtained by entering the keyword “Osteoporosis” from the DisGeNet database (https://www.disgenet.org/) [16]. Then, all the gene names were standardized and redundancy was deleted. Eventually, the obtained putative genes were used as the targets of OP.

### 2.4. Venn Diagram Analysis

Candidate targets of PA against OP were obtained by entered PA-related targets and OP-related targets into the Venn online tool (https://www.bioinformatics.com.cn/). The interaction of “PA-active compounds-target genes-OP” was constructed by Cytoscape software (version 3.7.2) [17].

### 2.5. PPI and Drug-Component-Target Network Construction

The above candidate targets were submitted to STRING (https://string-db.org/) [18] for protein-protein interaction (PPI) network construction, and only a confidence score of 0.7 was selected as the cutoff criterion. Cytoscape software (version 3.6.1) was used to visualize PPI network. Moreover, the most significant module of PPI network was found by the plug-in molecular complex detection (MCODE) for screening the clusters of original PPI network. Meanwhile, D-C-T network was also established by the calculation of Network Analyzer Plug-in in Cytoscape.

### 2.6. Gene Ontology (GO) and KEGG Pathway Enrichment

Last but not least, Metascape (https://metascape.org/gp/) [19], an online tool, was used to conduct GO enrichment and KEGG pathway analysis based on the above common target (min overlap = 3, *P* value cutoff = 0.01, and min enrichment = 1.5).

## 3. Results

### 3.1. Active Components of PA

A total of 14 candidate components were collected from BATMAN-TCM for further analysis as shown in Table 1.

### 3.2. The Potential Targets of PA against OP

To predict possible targets for PA, we imported the SMILES format of active components into SwissTargetPrediction, an online predictive tool, and a total of 320 targets of the 14 ingredients were identified. Then, the keyword “osteoporosis” was entered into DisGeNet database to predict 1098 targets associated with OP. Subsequently, 82 common targets were identified by generating a Venn diagram from the component-associated targets and OP-related targets, which were the potential therapeutic targets of PA against OP (Figure 1(a)). Using the 14 ingredients and the 82 common targets, a comprehensive view of the D-C-T network was formed (Figure 1(b)). The yellow circle represents the PA, the pink circle represents the active ingredient, and the blue diamond represents the targets. The results show that the active components with high degree of connectivity include Prostaglandin E1, 17-Beta-Estradiol, Alpha-Estradiol, and Estrone (≥15 gene targets).

RETRACTED

### 3.3. PPI Network and the Most Significant Module Analysis

Further searching for a key gene in PA against OP, the PPI network of 82 common targets was constructed (Figure 2(a)) and the most significant module was obtained using Cytoscape (Figure 2(b)). In the significant module, the top 5 nodal targets, including PIK3CA, MAPK1, ESR1, AKT1, and SRC, showed strong association with other proteins, suggesting higher degree for hubs. These hub proteins might have critical effects on the development of OP.

### 3.4. GO and KEGG Pathway Enrichment Analysis

In order to indicate the biological mechanisms of PA against OP, GO and KEGG pathway enrichment analyses of the 82 common targets were performed by using Metascape online tool. To gain insight into the specific functional characteristics, the 82 targets were categorized based on the following GO classes: biological process, molecular function, and cellular component. First, as depicted in Figure 3(a), the enriched biological process categories were dominated by response to peptide, cellular response to lipid, regulation of MAPK cascade, and so on. Second, cell component analysis showed that cell body and membrane raft mainly accounted for the largest proportion (Figure 3(b)). Finally, the enriched molecular function categories were dominated by lipid binding and hormone binding (Figure 3(c)).

In addition, the KEGG pathway analysis revealed that the 82 targets were mostly enriched in pathways in cancer and endocrine resistance (Table 2), such as estrogen signaling pathway, osteoclast differentiation, and HIF-1 signaling pathway.

## 4. Discussion

OP is mainly caused by the imbalance of bone formation and bone resorption [1, 2]. Traditional Chinese medicine has a long history of using PA in the treatment of OP, and the mechanism of action may involve multiple targets and pathways. PA has been reported to exert positive effects on chronic inflammatory and oxidative damages [6, 20, 21] as well as promote the proliferation and differentiation of many types of cells, including osteoblast and chondrocyte [6, 10, 22].

RETRACTED

For instance, Liu et al. found that PA can promote osteoblast differentiation and block TNF-*α*-mediated suppression of osteoblastogenesis via the NF-kB/p65 pathway as well as inhibit osteoclastogenesis in vitro [10]. Another study from Yun et al. suggested that PA promoted osteoblast proliferation, differentiation, and mineralization in vitro via the insulin signaling pathway, and the effect of PA on insulin signaling in osteoblasts may be mediated by the ERK pathway and the PI3K/Akt pathway [22]. Both the results indicated that PA could potentially be developed as an alternative treatment for OP. However, the understanding of specific mechanism through which PA against OP is still limited.

In the present study, network pharmacology based on various bioinformatics methods was used to examine the network of the molecular mechanisms of PA, and we first identified 14 active components of PA. Several of these components have been confirmed to have effect on bone metabolism. For example, estrogens, including estrone, Estrone, and 17-Beta-Estradiol, are key regulators of bone homeostasis. It is a consensus that estrogen deficiency has become an independent risk factor of postmenopausal osteoporosis (PMOP) [23–25]. Clinically, OP mainly occurs in postmenopausal women because the withdrawal of estrogen will cause excessive activation of osteoclasts, which disrupts the balance between normal bone formation and bone resorption. As a result, bone turnover is abnormally accelerated, which eventually leads to bone loss [26]. In addition, it has previously been reported that Prostaglandin E1 could stimulate the synthesis of osteoprotegerin (OPG), induce p38 MAP kinase phosphorylation, and strengthen osteoblast activation, which can significantly decrease BMD loss after liver transplantation and reduce the risk of bone fracture [27–29]. Most of the other active ingredients are also associated with osteoporosis, but it is worth noting that the relationship between Galactosamine and D-Galacturonic Acid and osteoporosis is not clear, and the effect of Retinol on bone metabolism varies with dose [30, 31]. Interestingly, previous studies found that Cholesterol, the active component of PA, was positively correlated with OP [32, 33]. However, Lecithin, another active ingredient, has been shown to lower blood lipid levels and increase bone density [34, 35].

The 82 common targets predicted from SwissTargetPrediction and DisGeNet database were found to be involved in both osteogenic and osteoclastic differentiation. Meanwhile, most of these common targets were hit by multiple ingredients at the same time, indicating that individual ingredients could act on the same targets, which finally played a synergistic effect in the treatment of osteoporosis. We carried out PPI network analysis, and the results show that the target proteins interact and regulate each other, rather than acting independently. The hub proteins, key targets for drugs to exert biological effects, especially PIK3CA, MAPK1, ESR1, AKT1, SRC, etc., have been confirmed to play an important role in the pathogenesis of OP [36–38]. Therefore, PA may act on these targets to improve bone mass and treat OP.

RETRACTED

GO analysis suggests that these common targets may play the function of lipid binding through subcellular structures such as cell body and membrane raft, thus participating in biological processes such as cellular response to lipid and regulation of MAPK cascade. As we know, when estrogen spreads to the nucleus, it binds to its nuclear receptor and regulates the transcription of downstream genes, which is closely related to behaviors such as lipid binding [24]. Moreover, KEGG pathway analysis also suggests that estrogen-related signal pathway may play a role in the treatment of OP by PA. Therefore, we speculate that PA may be effective in the treatment of OP by enhancing the binding of estrogen to its receptor. In addition, other signaling pathways, such as inflammatory mediator regulation of TRP channels (hsa04750) [39], neuroactive ligand-receptor interaction (hsa04080) [40], signaling pathway (hsa03320) [41], and GnRH signaling pathway (hsa04912) [42], are also involved in the regulation of bone metabolism and the pathogenesis of osteoporosis. However, these signaling pathways have not been reported in basic studies on the treatment of OP by PA. Therefore, our work suggested that there may be other signaling pathways besides the classic estrogen signaling pathways involved in the regulation of bone metabolism by PA.

Of course, there are limitations to our work, such as the lack of experimental validation of the results. In addition, the form and dose of PA depends on the doctor's experience and patient's situation, and there may be differences in efficacy and mechanism of action.

## 5. Conclusion

In general, this study revealed that mechanism of the anti-OP effect of PA is associated with the binding of estrogen. Predicting the effective components and action targets of PA through network pharmacology will help us to understand how PA affects bone metabolism and the potential molecular mechanism. Hence, it not only provides a pharmacological basis for clinical application of PA in treating OP but also gives us insight and inspiration for further research.

RETRACTED

## Figures and Tables

**Figure 1:** The potential targets of PA against OP. (a) Venn diagram of PA-related targets and OP-related targets. (b) “PA-active compounds-target genes-OP” network. Yellow circle: PA, pink circle: active ingredient, and blue diamond: targets.

**Figure 2:** PPI network and the most significant module analysis. (a) The PPI network from STRING was further analyzed using Cytoscape software. (b) The most significant gene was obtained using Cytoscape.

**Figure 3:** GO analysis. (a) Biological process analysis of 82 targets. (b) Cellular component analysis of 82 targets. (c) Molecular function analysis of 82 targets.

**Table 1:** Basic information of active compounds in PA.

PubChem CID	Name	Molecular structure
5870	Estrone	
5957	Adenosine Triphosphate	
5997	Cholesterol	
6042	Vitamin B1	
8815	Estragole	
24154	Galactosamine	
68570	Alpha-Estradiol	
161844	Lecithin	
439213	Glucosamine	
439215	D-Galacturonic Acid	
445354	Retinol	
5280723	Prostaglandin E1	
6918970	Estrone	
66795326	17-Beta-Estradiol	

**Table 2:** Top 10 in KEGG enrichment pathway analysis of 82 targets.

Pathway	Description	Count in gene set	LogP
hsa05200	Pathways in cancer	19/395	−16.312
hsa01522	Endocrine resistance	12/96	−15.343
hsa04750	Inflammatory mediator regulation of TRP channels	8/97	−8.881
hsa04080	Neuroactive ligand-receptor interaction	11/277	−8.638
hsa03320	PPAR signaling pathway	7/72	−8.333
hsa04912	GnRH signaling pathway	7/92	−7.582
hsa04657	IL-17 signaling pathway	7/93	−7.549
hsa00140	Steroid hormone biosynthesis	6/58	−7.372
hsa04931	Insulin resistance	7/107	−7.126
hsa04621	NOD-like receptor signaling pathway	8/170	−6.961

## Data Availability

The data used to support the findings of this study are available from the corresponding author upon request.
